The article "Assessing the Role of Nrf2/GPX4-Mediated Oxidative Stress in Arsenic-Induced Liver Damage and the Potential Application Value of Rosa roxburghii Tratt [Rosaceae]" was retracted in 2024. Reasons: signs of a paper mill; suspected computer-generated content; unreliable results or conclusions; concerns about the data.

# Assessing the Role of Nrf2/GPX4-Mediated Oxidative Stress in Arsenic-Induced Liver Damage and the Potential Application Value of Rosa roxburghii Tratt [Rosaceae]

**DOI:** 10.1155/2022/9865606

**Published:** 2022-04-25

**Authors:** Yuyan Xu, Qibing Zeng, Baofei Sun, Shaofeng Wei, Qingling Wang, Aihua Zhang

**Affiliations:** The Key Laboratory of Environmental Pollution Monitoring and Disease Control, Ministry of Education, School of Public Health, Guizhou Medical University, Guiyang 550025, China

## Abstract

Arsenic poisoning is a geochemical disease that seriously endangers human health. The liver is one of the important target organs for arsenic poisoning, several studies have shown that oxidative stress plays an important role in arsenic-induced liver damage. However, the specific mechanism of arsenic-induced oxidative stress has not yet been fully elucidated, and currently, there are no effective intervention measures for the prevention and treatment of arsenic-induced liver damage. In this study, the effect of the Nrf2/GPX4 signaling pathway and oxidative stress in the arsenic-induced liver damage was first evaluated. The results show that arsenic can activate the Nrf2/GPX4 signaling pathway and increase the oxidative stress, which in turn promotes arsenic-induced liver damage in MIHA cells. Moreover, when we applied the Nrf2 inhibitor, the promoting effect of arsenic on liver damage was alleviated by inhibiting the activation of the Nrf2/GPX4 signaling pathway. Subsequently, the Rosa roxburghii Tratt [Rosaceae] (RRT) intervention experiments in cells and arsenic poisoning population were designed. The results revealed that RRT can inhibit Nrf2/GPX4 signaling pathway to reduce oxidative stress, thereby alleviates arsenic-induced liver damage. This study provides some limited evidence that arsenite can activate Nrf2/GPX4 signaling pathway to induce oxidative stress, which in turn promotes arsenic-induced liver damage in MIHA cells. The second major finding was that Kaji-ichigoside F1 may be a potential bioactive compound of RRT, which can inhibit Nrf2/GPX4 signaling pathway to reduce oxidative stress, thereby alleviates arsenic-induced liver damage. Our study will contribute to a deeper understanding of the mechanisms in arsenic-induced liver damage, these findings will identify a possible natural medicinal food dual-purpose fruit, RRT, as a more effective prevention and control strategies for arsenic poisoning.

## 1. Introduction

Arsenic poisoning is a geochemical disease that seriously endangers human health [1], which can cause damage to multiple organs such as the skin, lungs, liver, and kidney [2]. The liver is one of the important target organs for arsenic poisoning, and hepatomegaly due to cirrhosis and ascites is its common clinical manifestation [3]. Previous studies [4, 5] have shown that the serum albumin (ALB), alanine aminotransferase (ALT), and total bilirubin (TBIL) are early biological markers reflecting liver damage in the arsenic poisoning population. And the oxidative stress caused by the decreased activity of antioxidant enzymes (such as superoxide dismutase (SOD), glutathione peroxidase (GSH-Px), and sulfhydryl (-SH)) and the increased production of lipid peroxidation product malondialdehyde (MDA) plays an important role in arsenic-induced liver damage. However, the specific mechanism of arsenic-induced oxidative stress has not yet been fully elucidated, and currently, there are no effective intervention measures for the prevention and treatment of arsenic-induced liver damage.

The article "Assessing the Role of Nrf2/GPX4-Mediated Oxidative Stress in Arsenic-Induced Liver Damage and the Potential Application Value of Rosa roxburghii Tratt [Rosaceae]" was retracted in 2024. Reasons: signs of a paper mill; suspected computer-generated content; unreliable results or conclusions; concerns about the data.

Nuclear factor E2-related factor 2 (Nrf2) is a key transcription factor regulating the cellular antioxidant defense system and plays an important role in defending against cellular oxidative stress [6–8]. However, increasing evidence [9] shows that environmental arsenic exposure can induce Nrf2-mediated adaptive antioxidant responses, which in turn regulate multiple antioxidant enzyme genes in vivo in response to oxidative and exogenous stress. Glutathione peroxidase 4 (GPX4) belongs to the glutathione peroxidase family and reduces lipid hydrogen peroxide to nontoxic lipid alcohols, thereby protecting cells from oxidative damage [10]. Several studies [11–13] show that GPX4 is regulated by Nrf2 and is an important transcriptional target of Nrf2. Therefore, study of the mechanism of oxidative stress from the perspective of NRF2/GPX4 signaling pathway is of great significance to better explain the cause of arsenic-induced liver damage. Moreover, finding natural medicinal food dual-purpose resources to inhibit oxidative stress and scavenge oxygen free radicals is also one of the important strategies to prevent and control arsenic poisoning.

Rosa roxburghii Tratt [Rosaceae] (RRT), a plant of the genus Rosaceae, is a unique wild resource in the Yunnan-Guizhou Plateau and the western Sichuan Plateau in China [14]. RRT contains a variety of rich nutrients and biologically active compounds, such as triterpenoids (the main ingredient is Kaji-ichigoside F1, and each gram of RRT contains about 0.176~0.183 mg of Kaji-ichigoside F1) and flavonoids [15]. Our previous animal study found that RRT can attenuate liver damage in arsenic-poisoned rats by inhibiting oxidative stress [16]. Other study [17] has also shown that RRT exhibit good hypoglycemic effects by activating the P13K/AKT signaling pathway and controlling hepatic gluconeogenesis and improving hepatic glycogen storage insulin resistance. However, little is known about the intervention mechanism of RRT and its potential application in the arsenic poisoning population.

The article "Assessing the Role of Nrf2/GPX4-Mediated Oxidative Stress in Arsenic-Induced Liver Damage and the Potential Application Value of Rosa roxburghii Tratt [Rosaceae]" was retracted in 2024. Reasons: signs of a paper mill; suspected computer-generated content; unreliable results or conclusions; concerns about the data.

In this study, we first observed the changes of oxidative stress (SOD, GSH-Px, -SH, MDA), Nrf2/GPX4 signaling pathway (Nrf2, GPX4), and liver damage- (ALB, ALT, TBIL) related indicators in the normal human liver cells (MIHA) exposed to arsenic and/or the Nrf2 inhibitor. Second, the RRT intervention experiments in cells and arsenic poisoning population were designed. By observing the changes in the above indicators, the aim was to study the mechanism and potential application value of RRT in arsenic-induced liver damage. Our study will contribute to a deeper understanding of the mechanisms in arsenic-induced liver damage, these findings will identify a possible natural medicinal food dual-purpose fruit that can be used to design more effective prevention and control strategies.

## 2. Materials and Methods

### 2.1. Study Population

According to the Standard of Diagnosis for Endemic Arsenism of China (WS/T 211-2015), a total of 92 arsenic poisoning patients (aged 30 to 65 yeas) were chosen from the Jiaole village, Xingren County, Guizhou Province, China, and were equally distributed to the RRT group (46 cases) and the placebo group (46 cases) by a block random design. In short, all participants first were divided into different block groups based on the gender and age (an interval every 5 years), and then, the same block group was equally distributed to the above two groups. The proposal of the intervention study protocol was reviewed and approved by the Ethics Committee of Guizhou Medical University (No. 201403001). All participants signed a written informed consent. All subjects must be local residents with a clear diagnosis of arsenic poisoning. Exclusion criteria included a recent history of seafood consumption and drugs (such as trace element supplements) that might affect arsenic metabolism.

RRT (the health food permission number of National Health Commission of the People's Republic of China is [2002]0004) and placebo were produced from the Sinopharm Group Guizhou Healthcare Industry Development Co., Ltd. Except the main component is glucose, the physical characteristics of the placebo (such as appearance, size, color, dosage form, weight, taste, and smell) are the same as those of RRT. Oral administration was used, with a dose of 20 mL each day (according to the recommended dosage in the health food instructions), once a day in the morning after breakfast for 90 days. During the entire cycle of the intervention, we performed a series of quality controls: (1) the entire study process was treated by full-time medical staff in Township Hospital Centers; (2) the regular monitoring and made daily records were conducted, including the food intake and intake habits of the participants, especially we strictly controlled the intake of seafood, trace element supplements, and preventive drugs for liver damage; and (3) the telephonic follow-up and on-site supervision were performed every day.

The article "Assessing the Role of Nrf2/GPX4-Mediated Oxidative Stress in Arsenic-Induced Liver Damage and the Potential Application Value of Rosa roxburghii Tratt [Rosaceae]" was retracted in 2024. Reasons: signs of a paper mill; suspected computer-generated content; unreliable results or conclusions; concerns about the data.

### 2.2. Questionnaire Interview and Sample Collection

A structured questionnaire was used to record the personal information of the subjects, such as demographic factors and health behavior. Fasting venous blood and hair behind the occiput (close to the hair root within 2 cm) was collected after obtaining informed consent from the study subjects, at both time points before the start of the intervention study and after the end of the intervention study. Hair arsenic content was measured using the hair behind the occiput, and the whole blood was used to detect the mRNA expression of the target gene, after extracting RNA. Non-anticoagulated blood samples were centrifuged at 3,000 g for 10 min at 4°C, and the serum was separated for the determination of oxidative stress, Nrf2/GPX4 signaling pathway, and liver damage-related indicators.

### 2.3. Cell Culture and Treatments

MIHA cells were purchased from the Global Bioresource Center of ATCC (USA), and the culture method was the same as described in the previous study [18]. Nrf2 inhibitor (ML385), Kaji-ichigoside F1, and sodium arsenite (NaAsO_2_) were purchased from Selleck (China), PUSH Biotechnology (China), and Merck (Germany), respectively. When MIHA cells in the logarithmic growth phase, the cells were collected and treated with 0, 5, 10, and 20 *μ*M NaAsO_2_ for 24 hours (h), according to the design of this study. In the part of the mechanism and the intervention study, the cells were treated with NaAsO_2_ for 24 h and then continued to intervene with the recommended concentration of ML385 (2.5 *μ*M) or Kaji-ichigoside F1 (10^−12^M) for 24 h. There were 4 groups which included the control group, NaAsO_2_ (20 *μ*M) treatment group, ML385 (2.5 *μ*M), or Kaji-ichigoside F1 (10^−12^M) treatment group, and NaAsO_2_ (20 *μ*M) combined with ML385 (2.5 *μ*M) or Kaji-ichigoside F1 (10^−12^M) treatment group. Each group had 3 complex holes, and the experiment was repeated 6 times.

### 2.4. Hair Arsenic Determination

Put the hair sample into the sample tube, and wash the hair sample with acetone (Merck, Germany), deionized water, deionized water, and acetone in sequence. After drying, use stainless steel scissors to cut the hair into approximately 1 mm segments to be measured. The determination of hair arsenic was described in previous studies [19]. In short, the inductively coupled plasma mass spectrometer (Avio 200, PerkinElmer, USA) was used for the determination of the content of arsenic in the hair. And the internal standard method and external standard method were used for quality control in the process of whole measurement. A trace element quality control sample (No. 8883 and 8884, Recipe, Germany) was added per 20 samples. For samples below the detection limit, we estimated the hair arsenic content to be half the detection limit.

The article "Assessing the Role of Nrf2/GPX4-Mediated Oxidative Stress in Arsenic-Induced Liver Damage and the Potential Application Value of Rosa roxburghii Tratt [Rosaceae]" was retracted in 2024. Reasons: signs of a paper mill; suspected computer-generated content; unreliable results or conclusions; concerns about the data.

### 2.5. Oxidative Stress Determination

All oxidative stress-related indicator kits were purchased from Nanjing Jiancheng Bioengineering (China). Following the protocol steps, as described in previous studies [20], hydroxylamine method was used for the determination of SOD, and microenzyme labeling for -SH, colorimetric method for GSH-Px, and TBA method for MDA. And the levels of the above indicators in cells were normalized by protein concentrations.

### 2.6. Enzyme-Linked Immunosorbent Assays

Human-specific Nrf2 and GPX4 were detected using the kits from Abcam (USA). The enzyme-linked immunosorbent assays were used for determining the concentration of Nrf2 and GPX4 in serum described as the previous study [18]. Each sample was designed in parallel and repeated 3 times, the mean absorbance was calculated to estimate the final concentration.

### 2.7. Liver Damage Indicator Determination

Serum ALB, ALT, and TBIL kits were purchased from BioSino Bio-Technology & Science, Inc. (China). After calibration and quality control, the serum concentration of the above indicators was determined as described in previous study [2], by an Olympus AU400 automatic biochemical analyzer (Japan). The levels of the above indicators in cells were determined according to the manufacturer's protocol, using the kits from BioAssay systems, which was described in previous study [21]. And the levels of the above indicators in cells were normalized by protein concentrations.

### 2.8. Quantitative Real-Time PCR

As described in the previous study [18], after the total RNA was isolated, the quantitative real-time PCR method was used to determine the levels of Nrf2, and GPX4 mRNA expression was determined according to the manufacturer's protocol, using the CFX96 Touch Deep Well Real-time PCR (Bio-Rad, USA). Table S1 shows the forward (F) and reverse (R) primer sequences of all genes which were synthesized by RiBoBio (Guangzhou, China). And the relative expression levels of Nrf2 and GPX4 were evaluated using GAPDH as an internal control. The primer sequences of all genes are presented in Table S1.

The article "Assessing the Role of Nrf2/GPX4-Mediated Oxidative Stress in Arsenic-Induced Liver Damage and the Potential Application Value of Rosa roxburghii Tratt [Rosaceae]" was retracted in 2024. Reasons: signs of a paper mill; suspected computer-generated content; unreliable results or conclusions; concerns about the data.

### 2.9. Western Blot Analysis

After the total proteins were extracted, the immune complex in PVDF membrane (Millipore, USA) was determined according to the manufacturer's protocol, using a chemiluminescence imaging system of Bio-Rad (ChemiDoc, USA), which was described in previous study [18]. The GAPDH was used as an internal control to assess the Nrf2, p-Nrf2, and GPX4 expressions and to normalize the blot. ALL antibodies were purchased from the Abcam (USA).

### 2.10. Statistical Analysis

The SPSS for windows version 22.0 software is used for the Kolmogorov-Smirnov test, Mann–Whitney *U* test, chi-squared test, *T*-test, one-factor analysis, and so on. For the results of cell experiments, the data were normally distributed, one-factor analysis was used to assess the difference of the oxidative stress, Nrf2/GPX4 signaling pathway, and liver damage-related indicators between the various groups, and the least significant difference test was used for further multiple comparisons. Demographic characteristic indexes and urinary arsenic were compared using chi-squared test and Mann–Whitney *U* test. The independent sample *T*-test was used to analyze the differences of the above indicators between the RRT group and the placebo group, before or after the intervention. And the paired *T*-test is mainly used to compare the differences of the above indicators before and after the intervention of various groups. Normally distributed data are expressed as mean ± standard deviation; otherwise, median and interquartile range will be used. The criterion for a significant difference was *P* < 0.05.

## 3. Results

### 3.1. Arsenite Can Activate Nrf2/GPX4 Signaling Pathway to Induce Oxidative Stress, Which in Turn Promotes Arsenic-Induced Liver Damage in MIHA Cells

To study the role of Nrf2/GPX4-mediated oxidative stress in arsenic-induced liver damage, the changes of oxidative stress (SOD, GSH-Px, -SH, MDA), Nrf2/GPX4 signaling pathway (Nrf2, GPX4), and liver damage- (ALB, ALT, TBIL) related indicators in the MIHA cells exposed to arsenic were observed. We sought to determine if Nrf2, GPX4 mRNA, and protein expression are regulated by arsenic, over a range of doses. After the treatment with 5 to 20 *μ*M NaAsO_2_, the expression levels of Nrf2 mRNA, protein and its phosphorylation expression were increased compared to the control group (*P* < 0.05). On the contrary, the GPX4 mRNA and protein expression were lower than the control group (*P* < 0.05). The above observed effect was more obvious in the 20 *μ*M NaAsO_2_ treatment group (*P* < 0.05). These results are presented in Figures 1(a)–1(c).

Figure 1(d) shows the effect of arsenic on oxidative stress. As illustrated in the figure, the concentration of SOD, GSH-Px, and -SH in the 5 and/or 10, 20 *μ*M NaAsO_2_ treatment groups is higher than that in the control group (*P* < 0.05), but the concentration of MDA in the 20 *μ*M NaAsO_2_ treatment group is lower than that in the 0 to 10 *μ*M NaAsO_2_ treatment groups (*P* < 0.05). And the dose-dependent relationship in the above indicators was more evident at the 20 *μ*M NaAsO_2_ treatment group (*P* < 0.05).

The article "Assessing the Role of Nrf2/GPX4-Mediated Oxidative Stress in Arsenic-Induced Liver Damage and the Potential Application Value of Rosa roxburghii Tratt [Rosaceae]" was retracted in 2024. Reasons: signs of a paper mill; suspected computer-generated content; unreliable results or conclusions; concerns about the data.

Subsequently, the early biological markers reflecting liver function were used to determine arsenic-induced liver damage. As revealed in Figure 1(e), the contents of ALT and TBIL in the 5 to 20 *μ*M NaAsO_2_ treatment groups were higher than the control group (*P* < 0.05), but the treatment of the MIHA cells with 5 to 20 *μ*M NaAsO_2_, the content of ALB was decreased compared to the control group (*P* < 0.05). Again, we found that the observed effect was most pronounced in the 20 *μ*M NaAsO_2_ treatment group (*P* < 0.05).

### 3.2. Inhibiting the Nrf2 Can Reduce the Oxidative Stress and Alleviates Arsenic-Induced Liver Damage in MIHA Cells

To examine if oxidative stress is regulated by Nrf2/GPX4 signaling pathway, we performed Nrf2 inhibitor experiments. The results indicate that the Nrf2 inhibitor ML385 can reduce the oxidative stress and alleviates arsenic-induced liver damage in MIHA cells (Figures 2(a)–2(e)), by downregulating the activation of the Nrf2/GPX4 signaling pathway. Figures 2(a)–2(c) clearly show that the expression of Nrf2 mRNA, protein and its phosphorylation expression was significantly reduced (*P* < 0.05), and the levels of GPX4 were significantly increased (*P* < 0.05) after the treatment with the ML385. As indicated in Figure 2(d), the concentrations of SOD, GSH-Px, and -SH in the NaAsO_2_ + ML385 group were higher than those in the arsenite-exposed group (*P* < 0.05), and the levels of MDA in the NaAsO_2_ + ML385 group were significantly decreased compared to those in the arsenite-exposed group (*P* < 0.05). Surprisingly, when we applied the Nrf2 inhibitor, the promoting effect of arsenic on liver damage was alleviated by inhibiting the activation of the Nrf2/GPX4 signaling pathway. As shown in Figure 2(e), the content of ALB in the NaAsO_2_ + ML385 group was higher than those in the arsenite-exposed group (*P* < 0.05). In contrast, the levels of ALT and TBIL in the NaAsO_2_ + ML385 group were significantly decreased compared to those in the arsenite-exposed group (*P* < 0.05).

### 3.3. Kaji-Ichigoside F1 Can Inhibit Nrf2/GPX4 Signaling Pathway to Reduce Oxidative Stress, Which in Turn Alleviates Arsenic-Induced Liver Damage in MIHA Cells

To understand the potential application value of RRT in the arsenic-induced liver damage, the main biologically active compound of RRT named Kaji-ichigoside F1 was used to perfume the intervention experiments in MIHA cells. Figures 3(a)–3(c) clearly show that the expression of Nrf2 mRNA, protein and its phosphorylation expression was significantly decreased (*P* < 0.05), and the levels of GPX4 were significantly increased (*P* < 0.05) after the treatment with the Kaji-ichigoside F1. Additionally, compared with the arsenite-exposed group, the concentrations of SOD, GSH-Px, and -SH in the NaAsO_2_ + Kaji-ichigoside F1 group were significantly increased (*P* < 0.05), and the level of MDA in the NaAsO_2_ + Kaji-ichigoside F1 group was lower than the arsenite-exposed group (*P* < 0.05) (Figure 3(d)). Surprisingly, the data shown in Figure 3(e) demonstrate that the content of ALB in the NaAsO_2_ + Kaji-ichigoside F1 group was significantly increased compared to the arsenite-exposed group (*P* < 0.05), and the levels of ALT and TBIL in the NaAsO_2_ + Kaji-ichigoside F1 group were lower than those in the arsenite-exposed group (*P* < 0.05).

The article "Assessing the Role of Nrf2/GPX4-Mediated Oxidative Stress in Arsenic-Induced Liver Damage and the Potential Application Value of Rosa roxburghii Tratt [Rosaceae]" was retracted in 2024. Reasons: signs of a paper mill; suspected computer-generated content; unreliable results or conclusions; concerns about the data.

### 3.4. RRT Can Inhibit Nrf2/GPX4 Signaling Pathway to Reduce Oxidative Stress, Thereby Alleviates Arsenic-Induced Liver Damage in Arsenic Poisoning Population

To advance translational applications of RRT (a natural medicinal food dual-purpose fruit), we sought to validate the effects observed in MIHA cells through a population intervention study. In this study, a total of 92 volunteers were included, and 83 subjects (including 40 cases in the RRT group and 43 cases in the placebo group) completed the standard and full-course intervention study, and the overall response rate was 90.22%.  Table 1 shows the characteristics of the study participants. Compared with the placebo group, the content of hair arsenic in the RRT group significantly increased (*P* < 0.05). There were no significant differences among the age, gender, smoking status, drinking status, and hair arsenic (before the RRT intervention) (*P* > 0.05).

Surprisingly, when we applied the RRT, the facilitation effect of arsenic on oxidative stress was significantly inhibited (Figure 4(c)) by reducing the activation of Nrf2/GPX4 signaling pathways (Figures 4(a) and 4(b)). More importantly, we also observed improvements in liver damage (Figure 4(d)). Figures 4(a) and 4(b) clearly show that the relative mRNA expression of GPX4 and the content of serum GPX4 in the RRT after intervention group were significantly increased compared with the placebo after intervention and the RRT before intervention groups (*P* < 0.05). In contrast, the relative mRNA expression of Nrf2 and the content of serum Nrf2 in the RRT after intervention group were lower than the placebo after intervention and the RRT before intervention groups (*P* < 0.05). The difference of oxidative stress-related indicators between various groups is presented in Figure 4(c). The contents of SOD, GSH-Px, and -SH in the RRT after intervention group were higher than those in the placebo after intervention and the RRT before intervention groups (*P* < 0.05). Compared with the placebo after intervention and the RRT before intervention groups, the content of ALB in the RRT after intervention group was significantly increased (*P* < 0.05), but the content of TBIL in the RRT after intervention group was significantly decreased (*P* < 0.05). These results are presented in Figure 4(d).

The article "Assessing the Role of Nrf2/GPX4-Mediated Oxidative Stress in Arsenic-Induced Liver Damage and the Potential Application Value of Rosa roxburghii Tratt [Rosaceae]" was retracted in 2024. Reasons: signs of a paper mill; suspected computer-generated content; unreliable results or conclusions; concerns about the data.

## 4. Discussion

Arsenic poisoning is a geochemical disease that seriously endangers human health [1]. Drinking water is the main exposure route worldwide [22, 23]. However, exposure to arsenic-contaminated diet and air via the burning of high-arsenic coal in unventilated indoor stoves is unique to China [24]. Guizhou province in southwest China used to be a typical area of arsenic poisoning, the arsenic content in coal can be as high as 35,000 ppm 20 years ago [25]. With the government's implementation to improve stoves, health education, etc., the total arsenic levels of coal fell to 8.35 ppm for median in 2017, and the diet, air in the region, and the urinary arsenic in the body have also been significantly decreased [24]. However, the cumulative and irreversible characteristics of arsenic poisoning on health, coupled with the unknown pathogenic mechanism of arsenic poisoning and the lack of effective therapeutic drugs, have become the bottleneck restricting the continuous control and elimination of the disease in the new era.

Oxidative stress refers to the imbalance between oxidation and antioxidant substances mediated by reactive oxygen species produced by the body, resulting in oxidative damage to tissue cells in the body [26]. Current research has shown that oxidative damage in the body is the basis for the pathogenesis of many diseases, and it is also one of the mechanisms common to the pathogenesis of many diseases in the body [27]. SOD is an important antioxidant enzyme in the first position of the oxidative stress defense system and can scavenge superoxide anion free radicals through reduction reactions and convert them into hydrogen peroxide, thereby blocking the chain reaction of free radicals and protecting cells from superoxide anion free radicals [28]. GSH-Px is also the most important antioxidant molecule in the body, which can catalyze the decomposition of hydrogen peroxide into nontoxic water molecules and can also catalyze the lipid peroxides formed in the peroxidation reaction [29]. The sulfhydryl in organisms mainly includes glutathione sulfhydryl and protein sulfhydryl, of which the former is the most important antioxidant sulfhydryl group of cells and plays an important role in antioxidation, protein oxidative damage repair, and amino acid transmembrane transport [30]. And the interaction of the above three antioxidant substances can remove free radicals in the body and block the chain reaction of free radicals, thereby protecting the body from oxidative damage by free radicals and reducing the production of lipid peroxidation product MDA [31]. Previous studies [32–36] observed arsenic exposure can cause the disruption of antioxidant defense systems. In this study, we also obtained the similar results, which indicated that arsenic could reduce the activity of antioxidant enzymes (such as SOD, GSH-Px, and -SH) and upregulate the concentration of the lipid peroxidation product of MDA. These findings provide more evidence of the association between arsenic exposure and oxidative stress. When we detect early biological markers of liver damage in cells, a surprising finding was that arsenic can significantly increase the concentration of ALT and TBIL and reduce the ALB. Our results provide more evidence for the hypothesis that ALB, ALT, and TBIL are early biological markers reflecting liver damage for arsenic exposure [8]. Furthermore, our findings are also suggestive of a link between oxidative and arsenic-induced liver damage because the recent studies [37, 38] have shown that the disruption of antioxidant defense system can cause damage to cells and tissues.

The article "Assessing the Role of Nrf2/GPX4-Mediated Oxidative Stress in Arsenic-Induced Liver Damage and the Potential Application Value of Rosa roxburghii Tratt [Rosaceae]" was retracted in 2024. Reasons: signs of a paper mill; suspected computer-generated content; unreliable results or conclusions; concerns about the data.

Nrf2 is a key regulatory mechanism for cells to resist oxidative stress to produce stress injury, which can control the expression of a series of antioxidant and detoxifying enzymes in cells, such as SOD, GSH-Px, and catalase [6, 7]. GPX4, a member of the glutathione peroxidase family, reduces the lipid hydrogen peroxide to nontoxic lipid alcohols, thereby protecting cells from oxidative damage [10]. An increasing number of studies [11–13] have shown that GPX4 is an important transcriptional target of Nrf2; however, studies on the role of Nrf2/GPX4 signaling in arsenic-induced liver damage by promoting oxidative stress are limited. Previous study has found that inorganic arsenic can activate the Nrf2 signaling pathway, which in turn regulates the expression of selenoproteins in mouse embryonic stem cells, such as GPX1 and GPX4. Our recent study showed that arsenic could be involved in arsenic-induced liver injury in rats by activating the PKC*δ*-Nrf2-ARE signaling pathway and promoting oxidative stress [39]. In this study, our results revealed that arsenite can activate Nrf2/GPX4 signaling pathway to induce oxidative stress, which in turn promotes arsenic-induced liver damage in MIHA cells. More importantly, when we applied the Nrf2 inhibitor, the promoting effect of arsenic on liver damage was alleviated by inhibiting the activation of the Nrf2/GPX4 signaling pathway. This finding provides evidence of the association between Nrf2/GPX4 signaling pathway-mediated oxidative stress and arsenic-induced liver damage. A large number of studies have shown that Nrf2 can play a role in maintaining the balance of redox state in body cells and reducing damage caused by oxidative stress [6, 7]. Our findings appear to be the opposite, a possible explanation for this finding may be that arsenic exposure may mediate cellular adaptive antioxidant responses by activating the Nrf2 signaling pathway, thereby aggravating oxidative damage-induced liver damage. Because increasing evidence [9] shows that environmental arsenic exposure can induce Nrf2-mediated adaptive antioxidant responses, which in turn regulate multiple antioxidant enzyme genes in vivo in response to oxidative and exogenous stress. The results of this study provide limited evidence supporting the hypothesis that arsenic can induce the body's adaptive antioxidant response by activating the Nrf2/GPX4 signaling pathway and promote oxidative stress, thereby aggravating arsenic-induced liver damage.

The article "Assessing the Role of Nrf2/GPX4-Mediated Oxidative Stress in Arsenic-Induced Liver Damage and the Potential Application Value of Rosa roxburghii Tratt [Rosaceae]" was retracted in 2024. Reasons: signs of a paper mill; suspected computer-generated content; unreliable results or conclusions; concerns about the data.

Recent studies [40] have shown that appropriate supplementation of vitamins, trace elements, and natural antioxidants can effectively reduce the health damage caused by arsenic exposure; particularly, the intervention of natural compounds or nutrients is considered a beneficial adjunctive treatment method for the detoxification of arsenic poisoning. RRT, a plant of the genus Rosaceae, is a unique wild resource in the Yunnan-Guizhou Plateau and the western Sichuan Plateau in China [14]. As the main active substance of RRT, Kaji-ichigoside F1 belongs to pentacyclic triterpenoids and has analgesic, anti-inflammatory, and antilipid peroxidation effects [14, 41]. In terms of liver damage, a previous study has shown that Kaji-ichigoside F1 exhibits hepatoprotective effects against d-galactosamine or lipopolysaccharide-induced liver damage in mice. The results of this study demonstrated that Kaji-ichigoside F1 can inhibit Nrf2/GPX4 signaling pathway to reduce oxidative stress, which in turn alleviates arsenic-induced liver damage in MIHA cells. To advance translational applications of RRT (a natural medicinal food dual-purpose fruit), we sought to validate the effects observed in MIHA cells through a population intervention study. A surprising finding was that RRT can inhibit Nrf2/GPX4 signaling pathway to reduce oxidative stress, thereby alleviates arsenic-induced liver damage in arsenic poisoning population. Moreover, hair arsenic is useful as an exposure biomarker, reflecting the arsenic intake of the chronic arsenic poisoning population [42]. Our results revealed that RRT significantly reduces arsenic levels in arsenic poisoning populations. A possible hypothesis is that RRT promotes arsenic excretion, which in turn exerts a protective effect against arsenic poisoning. However, we still need to provide more evidence to support this hypothesis. These results provide evidence that RRT can inhibit Nrf2/GPX4 signaling pathway to reduce oxidative stress, thereby alleviates arsenic-induced liver damage.

The article "Assessing the Role of Nrf2/GPX4-Mediated Oxidative Stress in Arsenic-Induced Liver Damage and the Potential Application Value of Rosa roxburghii Tratt [Rosaceae]" was retracted in 2024. Reasons: signs of a paper mill; suspected computer-generated content; unreliable results or conclusions; concerns about the data.

## 5. Conclusions

Overall, our study provides some limited evidence that arsenite can activate Nrf2/GPX4 signaling pathway to induce oxidative stress, which in turn promotes arsenic-induced liver damage in MIHA cells (Figure 5). The second major finding was that Kaji-ichigoside F1 may be a potential bioactive compound of RRT, which can inhibit Nrf2/GPX4 signaling pathway to reduce oxidative stress, thereby alleviates arsenic-induced liver damage (Figure 5). This study will contribute to a deeper understanding of the mechanisms in arsenic-induced liver damage, our findings will identify a possible natural medicinal food dual-purpose fruit, RRT, as a more effective prevention and control strategies for arsenic poisoning.

## Figures and Tables

**Figure 1:** Arsenite can activate Nrf2/GPX4 signaling pathway to induce oxidative stress, which in turn promotes arsenic-induced liver damage in MIHA cells. The in vitro results were based on 6 independent experiments. All data are presented as mean ± standard deviation. ^∗^, *P* < 0.05. (a) The relative mRNA expression of Nrf2 and GPX4. (b) The western blot for Nrf2, p-Nrf2, and GPX4. (c) The relative mRNA expression of Nrf2, p-Nrf2, and GPX4. (d) The concentration of oxidative stress-related indicators. (e) The content of liver damage-related indicators.

**Figure 2:** Inhibiting the Nrf2 can reduce the oxidative stress and alleviates arsenic-induced liver damage in MIHA cells. The in vitro results were based on 6 independent experiments. All data are presented as mean ± standard deviation. ^∗^, *P* < 0.05. (a) The relative mRNA expression of Nrf2 and GPX4. (b) The western blot for Nrf2, p-Nrf2, and GPX4. (c) The relative mRNA expression of Nrf2, p-Nrf2, and GPX4. (d) The concentration of oxidative stress-related indicators. (e) The content of liver damage-related indicators.

**Figure 3:** Kaji-ichigoside F1 can inhibit Nrf2/GPX4 signaling pathway to reduce oxidative stress, which in turn alleviates arsenic-induced liver damage in MIHA cells. The in vitro results were based on 6 independent experiments. All data are presented as mean ± standard deviation. ^∗^, *P* < 0.05. (a) The relative mRNA expression of Nrf2 and GPX4. (b) The western blot for Nrf2, p-Nrf2, and GPX4. (c) The relative mRNA expression of Nrf2, p-Nrf2, and GPX4. (d) The concentration of oxidative stress-related indicators. (e) The content of liver damage-related indicators.

The article "Assessing the Role of Nrf2/GPX4-Mediated Oxidative Stress in Arsenic-Induced Liver Damage and the Potential Application Value of Rosa roxburghii Tratt [Rosaceae]" was retracted in 2024. Reasons: signs of a paper mill; suspected computer-generated content; unreliable results or conclusions; concerns about the data.

**Figure 4:** RRT can inhibit Nrf2/GPX4 signaling pathway to reduce oxidative stress, thereby alleviates arsenic-induced liver damage in arsenic poisoning population. All data are presented as mean ± standard deviation. ^∗^, *P* < 0.05. (a) The relative mRNA expression of Nrf2 and GPX4. (b) The content of Nrf2 and GPX4 in serum. (c) The concentration of oxidative stress-related indicators. (d) The content of liver damage-related indicators.

**Figure 5:** Assessing the role of Nrf2/GPX4-mediated oxidative stress in arsenic-induced liver damage and the potential application value of RRT. Our study provides some limited evidence that arsenite can activate Nrf2/GPX4 signaling pathway to induce oxidative stress, which in turn promotes arsenic-induced liver damage in MIHA cells. The second major finding was that Kaji-ichigoside F1 may be a potential bioactive compound of RRT, which can inhibit Nrf2/GPX4 signaling pathway to reduce oxidative stress, thereby alleviates arsenic-induced liver damage.

**Table 1:** Characteristics of the study participants (*n* = 83).

Characteristics	Placebo (*n* = 43)	RRT (*n* = 40)	Statistical values	*P* values
Age	52.37 ± 7.39	53.95 ± 8.10	-0.93 ^1^	0.36
Gender			0.15 ^2^	0.70
Male	24 (55.81%)	19 (44.19%)		
Female	24 (60.00%)	16 (40.00%)		
Smoking status			1.53 ^2^	0.47
Never smoking	26 (60.47%)	19 (47.50%)		
Even smoking	13 (30.23%)	15 (37.50%)		
Now smoking	4 (9.30%)	6 (15.00%)		
Drinking alcohol status			0.56 ^2^	0.76
Never drinking	30 (69.77%)	26 (65.00%)		
Even drinking	10 (23.25%)	12 (30.00%)		
Now drinking	3 (6.98%)	2 (5.00%)		
Hair arsenic				
Before intervention	30.23 (17.66~37.79)	30.73 (23.64~39.85)	1.19 ^3^	0.28
After intervention	30.71 (15.60~46.48)	12.81 (10.57~17.00)	41.94 ^3^	<0.01

^1^ *T*-test, the statistical value is *T* value, the data were presented as mean ± standard deviation. ^2^Chi-square test, the statistical value is *χ*^2^ value, the data were presented as number (percentage). ^3^Mann–Whitney *U* test, the statistical value is *Z* value, the data were presented as median (interquartile range).

## Data Availability

The data supporting the conclusions of the study have been uploaded in the supplementary materials.

The article "Assessing the Role of Nrf2/GPX4-Mediated Oxidative Stress in Arsenic-Induced Liver Damage and the Potential Application Value of Rosa roxburghii Tratt [Rosaceae]" was retracted in 2024. Reasons: signs of a paper mill; suspected computer-generated content; unreliable results or conclusions; concerns about the data.

## Supplementary Materials

Supplementary 1 Supplementary table.pdf: the primer sequences.

Supplementary 2 Data.pdf: the data supporting the conclusions of the study.

## References

[1] Raju N. J. (2022). Arsenic in the geo-environment: a review of sources, geochemical processes, toxicity and removal technologies. *Environmental Research*.

[2] Zeng Q., Zou Z., Wang Q. (2019). Association and risk of five miRNAs with arsenic-induced multiorgan damage. *Science of the Total Environment*.

[3] Hsu L. I., Wang Y. H., Hsieh F. I. (2016). Effects of arsenic in drinking water on risk of hepatitis or cirrhosis in persons with and without chronic viral hepatitis. *Clinical Gastroenterology and Hepatology*.

[4] Jomova K., Jenisova Z., Feszterova M. (2011). Arsenic: toxicity, oxidative stress and human disease. *Journal of Applied Toxicology*.

[5] Zhou Q., Xi S. (2018). A review on arsenic carcinogenesis: epidemiology, metabolism, genotoxicity and epigenetic changes. *Regulatory Toxicology and Pharmacology*.

[6] Bellezza I., Giambanco I., Minelli A., Donato R. (2018). Nrf2-Keap1 signaling in oxidative and reductive stress. *Molecular Biology Reports*.

[7] Ma Q. (2013). Role of nrf2 in oxidative stress and toxicity. *Annual Review of Pharmacology and Toxicology*.

[8] Yao M., Zou Z., Zhang A. (2019). Association of endemic arsenic poisoning with liver injury: meta-analysis. *Chinese Journal of Endemiology*.

[9] Hu Y., Li J., Lou B. (2020). The role of reactive oxygen species in arsenic toxicity. *Biomolecules*.

[10] Forcina G. C., Dixon S. J. (2019). GPX4 at the crossroads of lipid homeostasis and ferroptosis. *Proteomics*.

[11] Dodson M., Castro-Portuguez R., Zhang D. D. (2019). NRF2 plays a critical role in mitigating lipid peroxidation and ferroptosis. *Redox Biology*.

[12] Kerins M. J., Ooi A. (2018). The roles of NRF2 in modulating cellular iron homeostasis. *Antioxidants & Redox Signaling*.

[13] Shin D., Kim E. H., Lee J., Roh J. L. (2018). Nrf2 inhibition reverses resistance to GPX4 inhibitor-induced ferroptosis in head and neck cancer. *Free Radical Biology & Medicine*.

[14] Shi C., Zhan L., Wu Y. (2020). Kaji-Ichigoside F1 and Rosamultin protect vascular endothelial cells against hypoxia-induced apoptosis via the PI3K/AKT or ERK1/2 signaling pathway. *Oxidative Medicine and Cellular Longevity*.

[15] Wu P. H., Han S. C., Wu M. H. (2020). Beneficial effects of hydroalcoholic extract from *Rosa roxburghii* Tratt fruit on hyperlipidemia in high-fat-fed rats. *Acta Cardiologica Sinica*.

[16] Xu Y., Yu C., Zeng Q., Yao M., Chen X., Zhang A. (2021). Assessing the potential value of Rosa roxburghii Tratt in arsenic-induced liver damage based on elemental imbalance and oxidative damage. *Environmental Geochemistry and Health*.

The article "Assessing the Role of Nrf2/GPX4-Mediated Oxidative Stress in Arsenic-Induced Liver Damage and the Potential Application Value of Rosa roxburghii Tratt [Rosaceae]" was retracted in 2024. Reasons: signs of a paper mill; suspected computer-generated content; unreliable results or conclusions; concerns about the data.

[17] Chen C., Tan S., Ren T., Wang H., Dai X., Wang H. (2022). Polyphenol from *Rosa roxburghii* Tratt fruit ameliorates the symptoms of diabetes by activating the P13K/AKT insulin pathway in db/db mice. *Food*.

[18] Zeng Q., Zhang A. (2020). Assessing potential mechanisms of arsenic-induced skin lesions and cancers: human and in vitro evidence. *Environmental Pollution*.

[19] Yang F., Yi X., Guo J. (2019). Association of plasma and urine metals levels with kidney function: a population-based cross-sectional study in China. *Chemosphere*.

[20] Wang Q., Wang W., Zhang A. (2021). TET-mediated DNA demethylation plays an important role in arsenic-induced HBE cells oxidative stress via regulating promoter methylation of OGG1 and GSTP1. *Toxicology In Vitro*.

[21] Amor C., Feucht J., Leibold J. (2020). Senolytic CAR T cells reverse senescence-associated pathologies. *Nature*.

[22] Podgorski J., Berg M. (2020). Global threat of arsenic in groundwater. *Science*.

[23] Rodriguez-Lado L., Sun G., Berg M. (2013). Groundwater arsenic contamination throughout China. *Science*.

[24] Wang D., Luo P., Zou Z. (2019). Alterations of arsenic levels in arsenicosis residents and awareness of its risk factors: a population-based 20-year follow-up study in a unique coal- borne arsenicosis county in Guizhou, China. *Environment International*.

[25] Finkelman R. B., Belkin H. E., Zheng B. (1999). Health impacts of domestic coal use in China. *Proceedings of the National Academy of Sciences of the United States of America*.

[26] Indo H. P., Yen H. C., Nakanishi I. (2015). A mitochondrial superoxide theory for oxidative stress diseases and aging. *Journal of Clinical Biochemistry and Nutrition*.

[27] Halliwell B. (2007). Oxidative stress and cancer: have we moved forward?. *The Biochemical Journal*.

[28] Zelko I. N., Mariani T. J., Folz R. J. (2002). Superoxide dismutase multigene family: a comparison of the CuZn-SOD (SOD1), Mn-SOD (SOD2), and EC-SOD (SOD3) gene structures, evolution, and expression. *Free Radical Biology & Medicine*.

[29] Taysi S., Tascan A. S., Ugur M. G., Demir M. (2019). Radicals, oxidative/nitrosative stress and preeclampsia. *Mini Reviews in Medicinal Chemistry*.

[30] Gorelenkova Miller O., Mieyal J. J. (2015). Sulfhydryl-mediated redox signaling in inflammation: role in neurodegenerative diseases. *Archives of Toxicology*.

[31] Czerska M., Mikolajewska K., Zielinski M., Gromadzinska J., Wasowicz W. (2015). Today's oxidative stress markers. *Medycyna Pracy*.

[32] Rahaman M. S., Akter M., Rahman M. M. (2020). Investigating the protective actions of D-pinitol against arsenic-induced toxicity in PC12 cells and the underlying mechanism. *Environmental Toxicology and Pharmacology*.

The article "Assessing the Role of Nrf2/GPX4-Mediated Oxidative Stress in Arsenic-Induced Liver Damage and the Potential Application Value of Rosa roxburghii Tratt [Rosaceae]" was retracted in 2024. Reasons: signs of a paper mill; suspected computer-generated content; unreliable results or conclusions; concerns about the data.

[33] Rahaman M. S., Banik S., Akter M. (2020). Curcumin alleviates arsenic-induced toxicity in PC12 cells *via* modulating autophagy/apoptosis. *Ecotoxicology and Environmental Safety*.

[34] Sener U., Uygur R., Aktas C. (2016). Protective effects of thymoquinone against apoptosis and oxidative stress by arsenic in rat kidney. *Renal Failure*.

[35] Souza J. M. O., Grotto D., Batista B. L., Junior Barbosa F. (2017). Distribution of arsenic and oxidative stress in mice after rice ingestion. *Journal of Trace Elements in Medicine and Biology*.

[36] Zhong G., Wan F., Yan H. (2020). Methionine sulfoxide reductases are related to arsenic trioxide-induced oxidative stress in mouse liver. *Biological Trace Element Research*.

[37] Rahaman M. S., Yamasaki S., Binte Hossain K. F., Hosokawa T., Saito T., Kurasaki M. (2020). Effects of curcumin, D-pinitol alone or in combination in cytotoxicity induced by arsenic in PC12 cells. *Food and Chemical Toxicology*.

[38] Susan A., Rajendran K., Sathyasivam K., Krishnan U. M. (2019). An overview of plant-based interventions to ameliorate arsenic toxicity. *Biomedicine & Pharmacotherapy*.

[39] Hu Y., Yu C., Yao M. (2018). The PKC*δ*-Nrf2-ARE signalling pathway may be involved in oxidative stress in arsenic-induced liver damage in rats. *Environmental Toxicology and Pharmacology*.

[40] Rahaman M. S., Rahman M. M., Mise N. (2021). Environmental arsenic exposure and its contribution to human diseases, toxicity mechanism and management. *Environmental Pollution*.

[41] Shi C., Li Z., Wu Y. (2020). Euscaphic acid and Tormentic acid protect vascular endothelial cells against hypoxia-induced apoptosis via PI3K/AKT or ERK 1/2 signaling pathway. *Life Sciences*.

[42] Hindmarsh J. T. (2002). Caveats in hair analysis in chronic arsenic poisoning. *Clinical Biochemistry*.

